This article has been retracted.

# Routine point-of-care ultrasound (POCUS) assessment of gastric antral content in traumatic emergency surgical patients for prevention of aspiration pneumonitis: an observational clinical trial

**DOI:** 10.1186/s12871-021-01357-y

**Published:** 2021-05-08

**Authors:** Mohamed S. Shorbagy, Amr A. Kasem, Ahmed A. Gamal Eldin, Ramy Mahrose

**Affiliations:** 1 Anesthesia and Intensive Care, Faculty of Medicine, Ain Shams University, Cairo, Egypt; 2 Diagnostic and Interventional Radiology Atomic Energy Authority, Faculty of Medicine, Ain Shams University, Cairo, Egypt

**Keywords:** Point of care, Gastric ultrasound, Emergency surgery, Polytrauma, Aspiration pneumonia

## Abstract

**Background:**

Polytrauma patients are at a higher risk of delayed gastric emptying. To assess the gastric volume, a reliable diagnostic tool is needed to prevent the occurrence of aspiration pneumonia, which remains a serious complication associated with anesthesia. Gastric antral ultrasound can provide reliable information about the size of the gastric antrum in traumatized patients undergoing emergency surgery.

**Methods:**

A prospective observational study of 45 polytrauma patients undergoing emergency surgery under general anesthesia was carried out. Prior to induction of anesthesia in the emergency department, gastric ultrasound was performed for qualitative and quantitative assessment of the gastric antrum in a supine position and right lateral decubitus (RLD) position. This was followed by routine placement of the nasogastric tube to aspirate and calculate the volume of the stomach contents.

**Results:**

Of the 45 polytrauma patients, the risk assessment of aspiration and the anesthesia technique changed in 14 patients (31.1%) after the gastric ultrasound examination.

A very good relationship existed between the expected stomach volume at the RLD position and the suction volume in the nasogastric tube. In all cases, no aspirations were documented.

**Conclusion:**

Ultrasound examination of the stomach in polytrauma patients allows assessing the size and type of stomach contents. The data obtained can influence the choice of anesthesia technique and reduce the risk of aspiration pneumonia.

**Trial registration:**

This trial was registered at ClinicalTrials.gov. registry number: NCT04083677 on September 6, 2019.

## Background

Pulmonary aspiration of gastric contents is rare in elective surgical groups but is more common in trauma patients requiring emergency surgery because trauma affects gastric motility and emptying [1].

The presence of residual gastric contents at the time of induction of anesthesia is an important risk factor of aspiration pneumonia. The routine use of bedside ultrasound provides valuable information about the volume and type of gastric contents. Preoperative gastric content determination helps the anesthesiologist to assess the risk of pulmonary aspiration [2, 3].

Ultrasonographic measurement of the antral cross-sectional area (CSA) may determine, based on the size of the stomach (i.e. the presence of solid particles and/or gastric volume < 1.5 ml/kg), the risk of occurrence of aspiration pneumonia during the perioperative period [4].

The aim of our study was to allow routine use of point-of-care ultrasound (POCUS) of gastric contents to assess aspiration risk and guide anesthetic management in trauma patients.

## Methods

A prospective observational study was conducted at the Ain Shams University Hospital Emergency Department. The approval of the Institutional Research Ethics Committee was obtained in August 2019 (approval number: FMASU R 42 / 2019). This study was registered on ClinicalTrials.gov (clinical trial ID NCT04083677) and carried out according to the Consolidated Standards of Reporting Trials (CONSORT) 2010 statement. It was conducted from September 2019 to January 2020. Written informed consent was obtained from all participants, or from the legal guardians for patients with a disturbed level of consciousness, before enrollment. The study included 45 polytrauma patients (18–65 years old of both sexes) admitted for emergency surgery.

The ABC protocol, the Glasgow Coma Scale (GCS) assessment, full laboratory and radiological examinations, and complete clinical assessment (including obtaining information about fasting hours) were carried out at the time of admission.

Exclusion criteria included pregnancy, history of upper gastrointestinal disorder, including gastroesophageal reflux disease, hiatal hernia, gastrointestinal cancer and/or upper gastrointestinal surgery, marked impaired level of consciousness (Glasgow Coma Scale less than 10), fractured base of the skull, and severe bleeding.

We used Siemens low frequency curved probe (2-5 MHz) and ACUSON × 300 ultrasound system from Siemens by an experienced radiologist as part of a focused assessment with sonography in trauma (FAST) studies. All patients were examined in the supine position, and then in the right lateral decubitus position (RLDP). The gastric antrum was determined at the level of sagittal scans in the epigastrium beneath the xiphoid and superior to the umbilicus. The liver (anteriorly), aorta, inferior vena cava and pancreas (posteriorly) were used as anatomical landmarks (Fig. 1).

**Fig. 1:** **a** Sagittal sonography of the gastric antrum. A = antrum; L = liver; P = pancreas; SMA = superior mesenteric artery; Ao = aorta. **b** Sagittal picture of the gastric antrum

The “empty” antrum appeared collapsed and “flat”, as the anterior and posterior walls were too close to each other (Fig. 2) or round to ovoid shape and resembled the target of a “bull’s eye” (Fig. 3).

**Fig. 2:** Sagittal sonogram of the empty antrum with a flat appearance. A = antrum; L = liver; P = pancreas; SMA = superior mesenteric artery; Ao = aorta

**Fig. 3:** Bull’s eye sign. L = liver; P = pancreas;. Ao = aorta

The antrum appeared to expand in a circle when it was filled with a transparent liquid (Fig. 4). Several gas bubbles appeared as punctuated hyper-echoic regions within the hypoechoic fluid, mimicking the formation of a “starry night” (Fig. 4a).

**Fig. 4:** **a** Sagittal sonography of the gastric antrum immediately following the ingestion of 200 mL of the clear fluid (“starry night” appearance). A = antrum; L = liver; P = pancreas. **b** Axial A = antrum, D = duodenum, Py = pylorus, IVC = inferior vena cava, Ao = aorta

The antrum with mixed echo contents appeared to expand when filled with solid contents, giving the film a “frosted glass” appearance (Fig. 5).

**Fig. 5:** Frosted glass sign. A = antrum; L = liver; P = pancreas; Ao = aorta

If the stomach contains clear liquids, volume measurement can help distinguish between a small volume that corresponds to baseline secretions and a larger volume than the baseline.

The antral cross-sectional area (CSA) was calculated after measuring the two antral dimensions [anteroposterior diameter (APD) and craniocaudal diameter (CCD)] according to the following equation: π [APD X CCD] / 4. The volume of the transparent fluid was calculated using the CSA measured in an RLD position and a previously published mathematical model: Volume (ml) = 27.0+ (14.6 x Right - Lat (CSA) - (1.28 x Age)). This equation accurately predicted the volume of the stomach, up to 500 ml [4].

Additionally, the antrum was classified according to a three-point rating system (Perlas score 0–2), based on the absence or presence of a clear liquid, in the supine and RLD position. Grade 0 indicates that there are no contents in the antrum in the supine and RLD positions. Grade 1 indicates a clear old liquid that can only be seen in the RLD position. Grade 2 indicates a clear liquid found in both the supine and RLD positions [3].

With explanations of the stomach ultrasound results and Perlas classification, we can plot this flowchart of risk stratification and decision-making (Fig. 6) [5].

**Fig. 6:** Flow chart of the analysis of the findings and medical decision-making based on the gastric point-of-care ultrasound

A nasogastric tube was inserted preoperatively to confirm gastric ultrasound volume calculation.

The low-risk class indicated a low risk of aspiration and it might be safe to perform surgery with slow induction of anesthesia by means of a laryngeal mask or endotracheal tube.

The high-risk class indicated a high risk of aspiration, with the following categories: 1, delay of surgery depending on its urgency (which might not be acceptable); 2, acid aspiration prevention medications such as metoclopromide and drugs that neutralize stomach acid such as non-particle antacids; H2 inhibitor and proton pump inhibitor; 3, nasogastric tube for gastric drainage; 4, local anesthesia and neuraxial anesthesia; and 5, general anesthesia with rapid sequence induction up to awake fibro-optic intubation.

### Primary endpoint

This included change in aspiration risk after gastric ultrasonographic assessment in comparison to clinical assessment.

### Secondary endpoints

These included the incidence of perioperative aspiration and the correlation between predicted volume in the RLD position and volume in the nasogastric tube.

#### Sample size calculation

The sample size calculation was performed, according to a study by Sabry et al. [6], to show the difference in change in aspiration risk of 45 patients after gastric ultrasonographic assessment in comparison to clinical assessment, with a confidence interval of 95%, acceptable margin of error of 5% and a power at 80%. The *p*-value was considered significant if < 0.05, and accordingly a minimal sample size of 45 patients was needed.

#### Statistical analysis

Analysis of data was done using IBM’s SPSS (Statistical Program for Social Science, version 16). The quantitative variables were described as means and standard deviations, while the qualitative variables were expressed as numbers and percentages. Statistical analysis was performed using statistical tests such as the Chi-square test, Student’s test, and table analysis. *P*-value < 0.05 was considered significant.

## Results

Forty-five polytrauma patients (25 males, 20 females) were scheduled for emergency surgery. Their demographic data are summarized in Table 1.

**Table 1:** Patient demographic data

Patient demographics	***N*** = 45
Gender M/F	25 (55.5%)/20 (44.4%)
Age (y) (mean and standard deviation SD)	40.22 ± 7. 11
Height (cm) (mean and standard deviation SD)	161.02 ± 1.13
Weight (kg) (mean and standard deviation SD)	80.65 ± 5.66
Body Mass Index (kg/m^2^) (mean and standard deviation SD)	31.88 ± 2.47

All data were presented as mean ± SD except gender which was presented as a percentage

Patients presented for various surgical procedures were showen in Table 2. The urgency of the operations was determined mainly from the surgical point of view.

**Table 2:** Surgical procedures performed

Surgical specialty	Number of the operations	Details of the operations
Neurosurgery	11	3 cases of compound depressed fractures, 1 case of extradural hemorrhage, 2 cases of subdural hemorrhage, 2 cases of lumbar fixation, 2 cases of cervical fixation and 1 case of intracerebral hemorrhage
Vascular surgery	9	4 cases of femoral vessel and 5 cases of brachial vessel exploration and repair
Orthopedics	11	5 cases of femur fracture fixation, 3 cases of humerous fracture fixation, 2 cases of fracture radius fixation and 1 case of fracture tibia fixation
General surgery	7	5 cases of abdominal explorations and 2 cases of deep wound repair
Plastic surgery	7	7 maxillofacial surgery

Detailed information about the types of intake and fasting intervals is provided in Table 3 (solid food intake *N* = 33, thick fluid *N* = 6, clear fluid *N* = 6; non-fasting *N* = 25, fasting *N* = 20).

**Table 3:** Clinical and gastric ultrasound assessment results and anesthetic decision-making plan changes

Patient number	Fasting duration/type of food intake	Anesthetic plan after clinical assessment	Gastric ultrasound			Anesthetic management after gastric ultrasound
			Type of content	Perlas grade	Conclusion	
1	4 h/bread and cheese	ETT: RSI	solid	–	Full	ETT:RSI
2	2 h/coffee	ETT: RSI	Empty	0	Empty	ETT: SI
3	6 h/banana	ETT:SI	Empty	0	Empty	ETT: SI
4	7 h/bread and cheese	ETT: SI	solid	–	Full	ETT: RSI
5	4 h/water	ETT: SI	Empty	0	Empty	ETT: SI
6	3 h/water	ETT: SI	Empty	0	Empty	ETT: SI
7	6 h/tea and biscuit	LMA	Empty	0	Empty	LMA
8	5 h/ vegetable soap	ETT:RSI	Empty	0	Empty	LMA
9	4 h/cheese sandwich with tea	ETT: RSI	solid	–	Full	ETT: RSI
10	2 h/water	ETT: SI	Empty	0	Empty	ETT: SI
11	2 h/coffee with milk	ETT: RSI	CF	II	Full	ETT: RSI
12	4 h/clear juice	ETT:SI	CF	1	Empty	ETT: SI
13	3 h/vegetable soap	ETT: RSI	Solid	–	Full	ETT: RSI
14	4 h/tea and water	ETT: SI	CF	I	Empty	ETT: SI
15	4 h/potato chips	ETT: RSI	solid	–	Full	ETT:RSI
16	3 h/bread and cheese with tea	ETT:RSI	Solid	–	Full	ETT:RSI
17	2 h/coffee and water	ETT:RSI	CF	II	Full	ETT:RSI
18	5 h/banana	ETT:RSI	Solid	–	Full	RSI
19	8 h/two meat sandwiches	ETT:SI	Solid	–	Full	ETT:RSI
20	8 h/mesh potato with rice	ETT:SI	Solid	–	Full	ETT:RSI
21	3 h/two cheese sandwiches and tea	Delay for 3 h	Solid	–	Full	Delay for 3 h
22	3 h/ bread and cheese	Delay for 3 h	Solid	–	Full	Delay for 3 h
23	6 h/ vegetable soap	ETT:SI	Solid	–	Full	ETT:RSI
24	4 h/cheese sandwich with tea	ETT:RSI	Solid	–	Full	ETT:RSI
25	2 h/water	ETT:SI	CF	II	Full	ETT:RSI
26	3 h/coffee with milk	Delay for 1 h	CF	II	Full	Delay for 1 h
27	3 h/clear juice	spinal	CF	II	Full	spinal
28	6 h/ vegetable soap	ETT:SI	Solid	–	Full	ETT:RSI
29	4 h/tea and water	ETT:SI	CF	II	Full	Delay for 2 h
30	4 h/potato chips	ETT:RSI	Solid	**–**	Full	ETT:RSI
31	5 h/ fried chicken	ETT:RSI	Solid	**–**	Full	ETT:RSI
32	4 h/ cheese sandwich	Delay for 2 h	Solid	**–**	Full	Delay for 2 h
33	9 h/ fatty meal	ETT:SI	Solid	**–**	Full	ETT:RSI
34	8 h/ meat and rice	ETT:SI	Solid	**–**	Full	ETT:RSI
35	8 h/ chicken	ETT:SI	Solid	**–**	Full	ETT:RSI
36	5 h/ rice and meat	ETT:RSI	Solid	**–**	Full	ETT:RSI
37	5 h/ fruits	ETT:RSI	Solid	**–**	Full	ETT:RSI
38	3 h/ meat	spinal	Solid	**–**	Full	spinal
39	3 h/ meat sandwich	ETT:RSI	Solid	**–**	Full	ETT:RSI
40	4 h/ pizza	Spinal	Solid	**–**	Full	spinal
41	9 h/ meat	ETT:SI	Empty	**0**	Empty	ETT:SI
42	8 h/ meat and potato	ETT:SI	Solid	**–**	Full	ETT:RSI
43	9 h/ rice with chicken	ETT:SI	Solid	**–**	Full	ETT:RSI
44	6 h/ fatty meal	Delay for 2 h	Solid	**–**	Full	Delay for 2 h
45	4 h/ 2 cheese sandwiches	Delay for 2 h	Solid	**–**	Full	Delay for 2 h

*CF* clear fluid, *ETT:RSI* Endotracheal intubation–rapid sequence induction, *ETT:SI* Endotracheal intubation–smooth induction, *LMA* Laryngeal mask airway

An empty stomach was documented in 10 patients (22.2%). The remaining 35 patients (77.7%) showed a full stomach on gastric sonography, where 29 of them had solid content and 6 had clear fluid of excess than 1.5 ml/kg. We found changed aspiration risk stratification and anesthesia decision-making in 14 patients (31.1%) following gastric ultrasound assessment, compared to preoperative clinical examination and fasting hour assessment (Fig. 7).

**Fig. 7:** Results of gastric ultrasound examination of gastric contents

Two patients (cases 2 and 8) were found to have a lower aspiration risk than anticipated by their history alone, and more liberal anesthetic techniques were used, as shown in the Table 3 and Fig. 8.

**Fig. 8:** Patient management

Twelve patients (cases 4, 19, 20, 23, 25, 28, 29, 33, 34, 35, 42 and 43) were found to have a higher aspiration risk than anticipated by thei history alone, and more conservative anesthetic techniques were used, as shown in Table 3 and Fig. 8.

As shown in Table 4, the number of patients with a high risk of aspiration increased after gastric ultrasonographic examination (from 25 to 35 patients), with the difference statistically significant. The number of patients with a low risk of aspiration decreased after gastric ultrasonographic examination (from 20 to 10 patients), with the difference statistically significant. This reflects the importance of routine point-of-care ultrasound (POCUS) assessment of gastric antral contents in traumatic emergency surgical patients for the prevention of aspiration pneumonitis.

**Table 4:** Change in aspiration risk after clinical assessment and gastric ultrasonography assessment

	After clinical assessment (*N* = 45)	After gastric ultrasonographic assessment (*N* = 45)	*P*-value
High risk of aspiration	25 (55.5%)	35 (77.7%)	0.0445^*^
Low risk of aspiration	20 (44.4%)	10 (22.2%)	0.0444^*^

All data were presented as percentages

*N* Number

^*^P-value < 0.05 = significant

Despite the fact that the statistical difference between the predicted volume in the RLD position and volume in the nasogastric tube was highly significant, a good clinical correlation was documented between them, as shown in Table 5.

**Table 5:** Correlation between predicted volume in the RLD position and volume in the nasogastric tube

**Predicted volume in RLD position (ml)** (mean and standard deviation SD)	200 ± 2.5
**Volume in the nasogastric tube (ml)** (mean and standard deviation SD)	190 ± 5.5
***P*-value**	< 0.001* HS

All data were presented as mean ± SD

*HS highly significant

## Discussion

Aspiration pneumonia remains a serious perioperative complication [7].

The presence of residual gastric contents at the time of induction of anesthesia is one of the major risk factors of pulmonary aspiration [8].

The motility of the digestive system can be affected by stress, pain, and anxiety, as well as by the use of opioids, which makes prediction of the gastric contents difficult. Patients with a “full stomach” were at a risk of aspiration during sedation or general anesthesia, as the tone of the lower esophageal sphincter and airway reflexes were reduced. The incidence of pulmonary aspiration was greater during emergency surgery [9].

The severity of aspiration was directly proportional to the volume, type and the acidity of the contents of the stomach. Because of basal gastric acid secretion, stomach volume less than 1.5 ml/kg was common in fasting patients and considered safe [7].

Data about fasting hours may be unreliable in elderly people with poor awareness, in children, and in cases of delayed stomach emptying, as in patients with multiple traumas who underwent emergency surgery [2].

In anesthesia, the use of gastric ultrasound provides more accurate information about gastric contents than the general assumption based on fasting hours [1].

Gastric ultrasound is a promising technology because it is readily available, non-invasive and relatively easy to use [10].

A retrospective study by Van de Putte et al. [11] indicated that gastric ultrasound might be a useful diagnostic tool, in addition to the standard assessment of gastric contents, if fasting guidelines were not followed in elective surgical patients. Also, this study revealed significant changes in aspiration risk stratification and anesthetic management following a standard history-based clinical assessment compared to an assessment based on gastric sonography in elective surgical patients who had not followed fasting guidelines.

We concluded, as Van de Putte et al. [11], that gastric ultrasound makes anesthetic management planning possible to prevent the risk of aspiration, but we allowed routine ultrasound for trauma surgical patients when the risk of aspiration was higher.

Bouvet et al. [4] reported the prevalence of a full stomach in 56% of emergency surgery patients and suggested that preoperative ultrasound assessment of gastric contents might be particularly helpful in such cases.

Sabry et al. [6] demonstrated that gastric ultrasound could be used as a reliable method to assess the residual gastric volume in fasting diabetics compared to the healthy control for elective surgery, and reported that the residual gastric volume in diabetic patients fasting for 8 h was higher than in patients without diabetes scheduled for elective surgery.

Cubillos et al. [2] concluded that bedside ultrasound could determine the type of gastric contents (nil, clear fluid, thick fluid or solid content). This qualitative information can be useful on its own to assess aspiration risks, especially in cases where the fasting state is unknown or uncertain.

In our study, we used gastric antral ultrasonography before induction of anesthesia in polytrauma patients undergoing emergency surgery to allow qualitative and quantitative assessment of the gastric antrum in supine and right lateral decubitus position for the prevention of aspiration pneumonitis.

Also, a nasogastric tube was inserted preoperatively to aspirate the gastric contents to be compared with gastric ultrasound volume calculation, with a very good correlation between them.

Our data suggest that routine gastric ultrasound in polytrauma patients allows the personalization of aspiration risk assessment to guide anesthetic management.

### Limitations

This study was subject to a number of limitations. Further studies with bigger sample sizes are needed to study and magnify the effect of gastric US in anesthetic management of polytrauma emergency patients, and to detect a larger number of patients with change in aspiration risk stratification. Also, studies with control groups are needed to fully support the results and conclusion by study data.

## Conclusion

We can conclude from this study that routine preoperative gastric ultrasound is a useful, safe and non-invasive tool for the assessment of gastric contents in emergency surgical patients, and for anesthetic management planning to prevent aspiration.

## Data Availability

The data sets used during the current study are available from the corresponding author on reasonable request.

## Abbreviations

POCUS: Routine Point of Care Ultrasound
RLD: Right lateral decubitus
CSA: Cross sectional area
CONSORT: Consolidated Standards of Reporting Trials
GCS: Glasgow Coma Scale
FAST: Focused assessment with sonography in trauma
A: Antrum
L: Liver
P: Pancreas
SMA: Superior mesenteric artery
Ao: Aorta
D: Duodenum
Py: Pylorus
IVC: Inferior vena cava
APD: Anteroposterior diameter
CCD: Craniocaudal diameter
SPSS: Statistical program for social science
CF: Clear fluid
ETT: RSI: Endotracheal intubation-rapid sequence induction
ETT: SI: Endotracheal intubation-smooth induction
LMA: Laryngeal mask airway
